RETRACTED

# Layout Optimization of Urban Cultural Space Construction Based on Forward Three-Layer Neural Network Model

**DOI:** 10.1155/2022/6558512

**Published:** 2022-06-03

**Authors:** Ye Zhou

**Affiliations:** Zhejiang University City College, Zhejiang, Hangzhou 310015, China

## Abstract

The change of urban cultural space layout is a multi-variable, multi-objective, and restricted research process. The optimization of urban cultural space construction and layout is a multi-objective decision-making problem that needs to be solved urgently. Based on the forward three-layer neural network theory, this paper constructs an optimization model for the construction and layout of urban cultural space evaluation of the layout of cultural space. This paper first analyzes the feasibility of combining the forward three-layer neural network model with the optimization and adjustment of cultural space layout structure. Taking the three-layer feedforward network as an example, the structure optimization model based on the forward three-layer neural network is selected, and the established model is used to reflect the internal environment of the objective world. Structure and perform dynamic simulation. In the process of simulation modeling, from the aspects of system description, model structure, logical analysis, reasoning, and interpretation, two effective computer dynamic simulation methods, namely, forward three-layer neural network model and system dynamics SD model, were carried out for theoretical comparison and identification. The experimental results show that the feasibility and calculation error of the application of the optimization model are relatively good, reaching 0.897 and 6.21%, respectively. The number of newly added cultural spaces and the expansion speed show an increasing trend, expanding at an average annual speed of about 35 km^2^, effectively increasing the quality of regional planning and construction layout.

## 1. Introduction

The formulation and implementation of the overall planning for cultural space layout are systematic projects. The formulation of the planning scheme is seriously affected by nature, society, economy, and other aspects. The technical method of cultural space layout planning has developed from early linear programming to multi-objective linear programming and even nonlinear planning, making the planning form develop from static planning to dynamic planning, and changing the original too rigid planning to the direction of flexible planning with certain adaptability [1–3]. Therefore, it shows the shortcomings of traditional planning methods, and it is very adaptable to the requirements of complex planning process. This requires the cultural space layout planning to adopt new theories and methods for the preparation and implementation management of cultural space layout planning according to the objective reality of the region and to deal with the relationship between the flexibility and rigidity of the planning, dynamic and static, so that the planning has more scientific operability [4–7]. For a certain area, there are many feasible urban planning schemes, and it is infeasible and unrealistic for us to find out these schemes one by one. At present, planners can only select candidate solutions based on qualitative methods. The selection process is called a “black box” operation. The results are subjective, and the number of solutions obtained is very small. In practice, there may be better solutions that have not been found, so it is necessary and urgent to seek an effective systematic method [8].

RETRACTED

Predictive analysis is an important part of cultural space layout planning, it is the premise and key to the success and failure of cultural space layout planning, and it is also a difficult problem in the research of cultural space layout planning [9–11]. Due to the complexity, nonlinearity, and uncertainty of the forecast data in the forecasting research of cultural space layout planning, traditional forecasting methods often fail. Therefore, on the basis of analyzing the modeling characteristics and problems of traditional forecasting methods, this paper introduces the cultural space layout planning forecasting method based on the forward three-layer neural network model and analyzes the neural network for establishing time series and regression analysis of two types of data. Taking the time series type as an example, the detailed technical design of the cultural space demand forecasting model based on the forward three-layer neural network is carried out, including network model selection, network structure design, sample construction, parameter setting, select the region and historical total population forecast as verification examples, establish a linear neural network model of population forecast for simulation forecasting, to verify the forecasting ability of the forward three-layer neural network model, and compare and analyze the artificial neural network Similarities and differences between network prediction models and traditional prediction methods [12–14].

Therefore, from the perspective of model methodology, this paper takes the preparation stage of the overall planning of cultural space layout at the micro-level as the starting point and analyzes mode. The neural network method is combined with the overall planning technology of cultural space layout, based on the theoretical analysis of the cultural space layout planning model method based on the forward three-layer neural network model. On the basis of introducing the theoretical development and principle of the forward three-layer neural network, the three most important feedforward types, such as the forward three-layer neural network model, the radial basis function (RBF) network model, and the linear neural network model, are analyzed emphatically. The neural network model is discussed. Through systematic analysis of land use structure, necessary knowledge is obtained, samples of land use structure change are extracted, existing samples are studied, trained, and tested, and artificial neural network dynamic simulation model is established. The network structure, mathematical description of the algorithm, and the setting of learning parameters are discussed for these three models. The advanced algorithm and neural network toolbox for high-performance numerical computation of MATLAB software are laid out, the realization process of artificial neural network model based on MATLAB software is expounded, and the realization method of GIJI based on MATLAB and the realization method of M language programming are discussed in detail. Take the region as an example to verify the region, establish a forward three-layer neural network model for cultural space layout planning in a new round of special research on the revision of the overall planning of regional cultural space layout, and systematically carry out planning practice problems based on the forward three-layer neural network model.

RETRACTED

## 2. Related Work

The analysis of the traditional planning model method can fully show that the existing traditional planning model method is limited to emphasizing the deterministic functional relationship between the planning elements, and it is a method based on reasoning step by step. It is difficult to modify, and it is also difficult for the model results to dynamically reflect the changes of the plan in real time. Effective dynamic planning cannot be carried out, and it is impossible to realize the flexible planning scheme of cultural space layout planning. To achieve dynamic planning or flexible planning, it is necessary to rebuild the model, set the model parameters, and re-run the operation. Model theoretical comparison is combined with model empirical comparison [15–17].

Moustafa et al. [18] believed that, with the construction of the forward three-layer neural network model for cultural space layout planning as the main line, in the research on the optimization of cultural space layout structure, theoretically identify and compare the forward three-layer neural network model and the system dynamics SD model. In terms of cultural space demand forecast and cultural space layout planning evaluation research, Song et al. [19] analyzed it separately, combined with other main model methods to conduct empirically combined analysis to confirm the effectiveness of the neural network model for cultural space layout planning. Encouraged by the achievements of systems engineering technology in solving complex engineering problems, Liu et al. [20] began to apply systems engineering technology and computer technology to urban development research and applied the knowledge of systems theory and synergy theory in the research process; it is used to coordinate the relationship between the expansion of urban construction land and factors such as transportation, infrastructure layout, and greening. However, in the actual process, these studies excluded public participation and failed to produce the expected effect on urban development, so they were met with huge doubts and censures.

RETRACTED

While evaluating and predicting the cultural space capacity and service capacity, through GIS technology, the urban cultural space is divided into several categories, and then the method of detailed investigation is used to determine the mixing degree and building density of the future cultural space layout. Development needs are forecasted and simulated. In terms of the driving force mechanism of urban construction land expansion, Wang et al. [21], from the perspective of the dynamics of urban spatial structure changes, comprehensively used economics and sociology to analyze and proposed three models that affect the city: the combined force model, the coverage model, and integrated models. Sun and Lei [22] pointed out that there are four driving forces for urban space expansion: the driving force of economic development, the market force of cultural space, the driving force of the development of transportation and communication facilities, and the driving force of population growth. At the same time, we believe that natural factors, ecological environment factors, location factors, social and cultural psychology, and behavior patterns can also have a huge impact on urban construction land. Cheng believes that for mountain cities, natural topography is a key factor affecting urban spatial expansion [23–25]. The researchers also discussed that the generation and transformation of modern means of transportation are also the important driving forces for the generation and development of modern cities. Residential diffusion plays a very important role in the expansion of cities to the periphery. Therefore, some researchers focus on considering the influence of single factors such as traffic and residential on the expansion of urban space.

RETRACTED

## 3. Layout Optimization of Forward Three-Layer Neural Network Model

### 3.1. Forward Three-Layer Neural Network Nesting

In the forward three-layer neural network target decision, *P* and *q* are generally a function of a certain attribute of the thing, that is, the possibility and satisfaction of the attribute of the thing. Different attributes *r* and *s* of things can be selected according to needs, so as to obtain the possibility function *P*(*r*) and the satisfaction function *q*(*s*).

(1) $$\begin{array}{c} \sum_{i+j=c}^{i}{\left(-t\right)}^{i-1}k\left(t-1\right)-\sum u{\left(t\right)}^{j}\\ =\sum_{i+j=c}^{i}{\left(-t\right)}^{i-1}k\left(t-1\right)-{\sum k\left(u\right)}^{j}. \end{array}$$

They can be continuous functions or discrete functions. Generally, in practical decision-making, try to simplify the functional form of Figure 1, and use a three-fold curve or an *S*-shaped curve to describe the change of likelihood or satisfaction from 0 to 1. Evaluating the cooperative performance of individuals in various groups according to the cooperative relationship (or cooperative fitness value, taking the fitness value of the complete solution as the evaluation index), adopt appropriate strategies to extract typical individuals of various groups.

In steady state, the total flux through the control volume is zero; that is, flux equilibrium is reached. The way of deriving discrete equations by the finite volume method is based on the integral equation of the control volume, which is essentially different from the derivation process of the finite difference method. In addition, each term in the discrete equation has its own definite physical meaning, which also determines that the finite volume method has more advantages than the finite difference method and the finite element method.

(2) $$\begin{array}{c} x_{a-b}^{a+b}\left(t,t-1\right)-x_{a-b}^{a+b}\left(1-a{\left(t\right)}^{2}-b{\left(t-1\right)}^{3}-c\right)=0. \end{array}$$

For a forward three-layer neural network, there is a probability curve *P*(*r*) for one attribute *r* and a satisfaction curve *Q*(*s*) for another attribute *S*, and *r* and *s* satisfy a certain relationship with the attribute a. That is, the limiting conditions *F*(*r*, *s*, *a*), *P*(*r*), and *Q*(*s*) can be combined into a possible satisfaction curve relative to the attribute a through certain rules, which quantitatively describes the degree of both possible and satisfactory, denoted as *w*[0,1]. When *w*=1, it is 100% possible and satisfactory; when *w*=0, it is completely impossible or completely dissatisfied or neither completely possible nor completely satisfactory.

RETRACTED

### 3.2. Neural Network Training Process

In the neural network, the storage of knowledge and information is represented as a distributed physical connection between neurons, which is distributed and stored in each neuron and its connections in the entire network. Each neuron and its connections only represent a part of the information, rather than a complete specific concept. Specific concepts and knowledge can only be expressed through the distributed combined effect of each neuron. Due to the large number of neurons in the forward three-layer neural network and the huge information storage capacity of the entire network, it has a strong ability to process uncertain information. Even if the input information is incomplete, inaccurate, or ambiguous, the neural network is still able to associate the complete picture of the thing in the memory.

Supervised learning is what we commonly use and needs to be based on a certain number of samples. The network in Figure 2 will automatically compare the actual output with the ideal output and then adjust the weights according to a specific algorithm. This process continues to cycle until the accuracy is satisfied until the request is set. Among them, the most commonly used algorithm is delta rule incremental learning.

(3) $$\begin{array}{c} r\left(s,t\right)=\frac{L\left(s,t\right)}{\sqrt{s\left(t,1\right)-t\left(s,1\right)}}-\frac{L\left(s^{\prime },t^{\prime }\right)}{\sqrt{t\left(s^{\prime },1\right)-s\left(t^{\prime },1\right)}}-1. \end{array}$$

The most commonly used turbulence models are mainly divided into Reynolds stress model and viscous model. The following is only a brief introduction. Reynolds stress model includes Reynolds stress equation model and algebraic stress equation model. This model directly establishes Reynolds stress equation and replaces the right end of the equation. It is the characteristic scale expression of average flow and turbulent flow. Although it can reflect the variation law of Reynolds stress with time and space, it has a large amount of calculation and high computer requirements, so it is not as widely used as the eddy-viscous model.

### 3.3. Input of Urban Culture Samples

The objectives of most cultural spatial layout optimization configurations are multi-objective. When constructing a multi-objective planning model, two principles should generally be followed, that is, the principle of “reducing more to less,” that is, on the premise of meeting the planning needs, conduct a comprehensive analysis and minimize the number of objectives.

(4) $$\begin{array}{c} \left\{\begin{array}{c} y\left(t,t+1\right)=\left(1+t\right)y\left(t-1,1\right),\\ x\left(t,t+1\right)=\left(1-t\right)x\left(t,1\right). \end{array}\right. \end{array}$$

Common methods include eliminating subordination, are necessary for less specific goals, combine several similar goals, and turn secondary goals into constraints. Secondly, the goals can be sorted. When selecting the plan, the important goals are first considered, those plans that cannot meet the important goals are eliminated, and then the secondary goal selection plan is considered.

RETRACTED

Figure 3 uses a master forward network cluster and several slave forward network clusters. Each slave forward network cluster evolves independently. After each iteration, the best particles are copied to the master forward network cluster, then the master forward network cluster begins to evolve, finds the best particle, and feeds this particle information to each slave forward network cluster, and then each slave forward network cluster modifies the speed of the particle according to this information and continues to evolve. Each slave forward network cluster exchanges information through the master forward network cluster, and the information exchange process of each forward network cluster is shown in the text. In this way, the excellent individuals of each subgroup can be selected and retained, and the evolution speed can be accelerated while maintaining the stability of the evolution of the excellent individuals, so as to avoid the premature convergence phenomenon in the evolution of a single group.

(5) $$\begin{array}{c} \frac{\exp\left(t\right)-n\left(1\right)}{\exp\left(t\right)+n\left(1\right)}=\frac{n\left(x\right)\exp\left(a+bt\right)}{\exp\left(t\right)}. \end{array}$$

The evolution process of each slave population adopts the mixed algorithm—GSO algorithm; that is, one part of the slave forward network cluster adopts the algorithm to perform crossover and mutation operations, and the other part adopts the algorithm to update the speed and position according to the speed and position. The master forward network cluster adopts an algorithm, which is updated according to the speed and position. In this way, the excellent individuals of each sub-forward network cluster can be selected and retained, while maintaining the stability of the evolution of the excellent individuals, speeding up the evolution speed and avoiding the premature convergence phenomenon in the evolution process of the single forward network cluster.

### 3.4. Output of Spatial Construction Layout Results

With the support of GIS spatial construction and layout technology, various related planning maps, cultural space suitability evaluation maps, and current land layout maps are stacked together, and common area boundaries are determined according to the overlapping situation. All overlapping and basically overlapping boundaries can be directly used as the boundaries of cultural space layout divisions; for nonoverlapping parts, the dominant future use of this part of cultural space should be analyzed. More similar, merge this part of the cultural space into that use area.

(6) $$\begin{array}{c} g\left(i,j\right)=\left\{g_{i-1,j-1}^{1,1},g_{i-1,j-1}^{1,2},g_{i-1,j-1}^{1,3},\ldots ,g_{i-1,j-1}^{1,i-j},\ldots ,g_{i-1,j-1}^{1,i+j}\right\}. \end{array}$$

In the specific operation, the overlay model can integrate the agricultural zoning map and the urban planning map, focusing on the cultural space suitability evaluation map, and then refer to other planning and zoning maps for zoning. If it is necessary to change the originally approved planning boundary when dividing the area for use, great care should be taken, and the reason for changing the boundary should be explained in consultation with the original planning department. The model in Table 1 is suitable for areas where various planning and zoning maps are relatively complete.

RETRACTED

The processing method used in this paper is the standard wall function method, which has a better simulation effect in engineering practice. The variables in the core area are correlated, so that the variable values of the nodes on the control volume adjacent to the wall can be obtained. The selection of the number of hidden layer nodes has always been an important issue in the optimization of the forward three-layer neural network. If the number of nodes is too small, the network may not be trained, or the trained network is not strong enough to recognize the samples that do not appear; that is, the fault tolerance is very poor, and it is easy to fall into local minima, which will affect the accuracy of network learning and adverse effects; if the number of nodes is too large, the generalization ability of the network will be reduced, making it difficult to adapt to new inputs, and at the same time, the training time may be too long, and the error may not be optimal.

## 4. Construction of an Optimization Model for Urban Cultural Space Construction Layout Based on Forward Three-Layer Neural Network

### 4.1. Forward Three-Layer Neural Network Interconnection

This paper compares SA-MPSC algorithm and simple algorithm based on simulated forward network cluster, multi-particle swarm co-evolutionary algorithm (MPsc), three kinds of Rosenbrock function (*f*1), RaSt^n function (rubbish), and Griewank function (*f*3). In the process of optimization, the curve of MPSC is smoother than that of MPSC, and there is no obvious jump, while the curve of MPSC is somewhat jumpy, which shows SA. The ability of MPSC to coordinate and balance the layout and global exploration is stronger than that of MPSC, and the new and excellent experience of exploration can be deployed in time. Moreover, with the passage of time, the gap between SA-MPSC and MPSC in the continuous evolution ability has a gradually increasing trend. That is, in the later optimization process of various group evolutions, the fitness value of each individual in various groups accepts the optimal solution according to the metropolis acceptance criterion and at the same time the probability accepts the deteriorating solution.

RETRACTED

It can be seen that, except for individual points, most of the output errors of the samples in Figure 4 are below 5%, and after learning, the error of the comparison group is about 4%, indicating that the network is well trained and can be used to predict any input.

(7) $$\begin{array}{c} 1-\frac{1-d\left(i,j\right)}{d\left(1\right)+d\left(2\right)+\cdots +d\left(i\right)}-\frac{d\left(i\right)d\left(j\right)}{d\left(1\right)+d\left(2\right)+\cdots +d\left(j\right)}-\cos\left(i\right)\cos\left(j\right)=1. \end{array}$$

The network has two layers, and the input data have 24 dimensions, so the number of neurons in the input layer is *m* = 24; the neurons in the competition layer are distributed in a two-dimensional array (*S* rows, *S* columns, *S*2 in total), and the number represents the potential of the input data. Since the number of categories is unknown, and the number of neurons in the competition layer is generally much more than the number of categories, this paper takes the number of neurons in the competition layer *S*2 = 9, 16, 25 and conducts network learning, respectively, so that the same type of winning neuron is given. The abundant response field also makes the separation of various types of neurons obvious, and the clustering results have better visualization effect as in the text. This phenomenon shows that the ability of utilization to coordinate and balance with global exploration is stronger than MPSC, and the new and excellent experience of exploration can be utilized in time. And with the passage of time, the gap between SAC and MPSC in the ability of continuous evolution tends to gradually increase.

(8) $$\begin{array}{c} \sum_{i,j}x\left(i,j\right)\frac{\mathrm{cov}\left|x\left(i\right)-\left(j\right)\right|}{\mathrm{cov}\left|x\left(i\right)\right|-\mathrm{cov}\left|x\left(j\right)\right|}-1=0. \end{array}$$

In the SA-MPSC and MPSC algorithms, each particle is set to 10 dimensions, and the number of subgroups in the particle group is *M* = 6; the number of forward three-layer network nodes in each subgroup is *m* = 20, and the corresponding main group in the forward three-layer network. The number of nodes *m* is 6; in each iteration of the algorithm, the forward three-layer network nodes in each subgroup are divided into two groups according to the probability of 0.5: one group operates according to the update speed and position of the formula, and the other is the group operate; when the main group operates, the speed and position of the forward three-layer network nodes are updated according to the formula, and the inertia weight also varies from 0.7 decrements to 0.3, learning coefficient *C*-ma. The value of *t* − *e* is the same as that of the subgroup.

RETRACTED

### 4.2. Evaluation of Urban Cultural Data

The urban cultural data of the four-layer network are easier to enter the local minimum than the three-layer network, so the three-layer network with only one hidden layer can be used. As for the topology design of the three-layer forward three-layer neural network, the basic connection method can be used; that is, the nodes of the two adjacent layers are fully connected to each other. A better accuracy can be obtained within the system, and there can also be direct connections between the nodes of the input layer and the nodes of the output layer. Take BP as an example to design a forward three-layer neural network model for cultural space layout planning, and design a forward three-layer neural network model for cultural space demand forecasting, a forward three-layer neural network model for cultural space layout structure optimization, cultural space layout planning, and scheme evaluation forward three-layer neural network model.

The forward three-layer neural network model design of cultural space demand forecast only takes time series data as an example, while the design of regression analysis prediction model is similar to the design of cultural space layout structure optimization model. The number of nodes in the output layer is 1. Initially, samples 5 and 6 are used for testing samples, and samples 1 to 6 are used for learning samples. After passing the test, samples 5 and 6 are added to the ranks of learning samples for re-learning and training of the linear neural network.

When the first form is used, the sample input of the forward three-layer neural network and the output of Figure 5 are completely independent variables, which will reduce the prediction ability of the network; while the second form uses the time series as a reference, considering the sample input and the correlation effect between the outputs can better capture the change trend of the time series. Practice has proved that the prediction effect of using the second form to determine the sample of the forward three-layer neural network prediction model is better than that of the first form.

(9) $$\begin{array}{c} \frac{\left(1-x\left(t\right)-t\right)\text{d}x\text{d}t}{x\left(t\right)\text{d}x}-\frac{ax\text{d}x}{1-btdt}=u\left(x\right)\text{d}u\text{d}x. \end{array}$$

The neural network can trend to extrapolate the mastered rules to adapt to the unknown model. The method is that the model established according to a set of sample data can be used for the prediction of nonsample data. For time series data, using a set of samples or partial data to train and achieve convergence, the model has the ability to predict nonsample data and is a prediction of future unknown data. For the input of each network, only a part of the weights are adjusted to make the weight vector more deviated from or closer to the input vector. This adjustment process is competitive learning. With continuous learning, the ownership vectors are separated from each other in the input vector space, thus forming that each represents a class of patterns in the input space, which is the clustering function of automatic feature recognition of the SOM network.

RETRACTED

### 4.3. Distribution of Spatial Construction Layout Indicators

Layout index regression analysis, also known as correlation analysis, is the most effective method to analyze and predict the causal relationship by analyzing the quantitative form of the mutual influence and mutual restriction relationship that may exist between variables. There is a causal relationship between a large number of variables in her layout planning, but we often cannot grasp the causal relationship between them or cannot clearly and accurately state the quantitative law of their causal relationship, but only from statistics, accumulate their quantitative performance during sampling. Regression analysis explores the relationship between variables through the process of hypothesis, parameter estimation, and verification. Taking the state equation as the core of the model algorithm, the decision equation, auxiliary equation, and initial equation are the main contents of the state equation, and the state variable, auxiliary variable, and rate variable are its key variables.

(10) $$\begin{array}{c} x_{i}^{i-1}\left(t\right)=\frac{x\left(t\right)-x_{i}^{1-t}}{x_{i}^{i-1}}-\frac{x\left(t\right)-x_{i}^{2-t}}{x_{i}^{i-1}}-\cdots -\frac{x\left(t\right)-x_{i}^{n-t}}{x_{i}^{i-1}}-1. \end{array}$$

The meaning and goal of the persimmon problem are different for the reliance of the bait. For gate array mode and forward network cluster placement, the layout problem becomes an allocation problem, where the goal is to achieve a high cat pass rate; for standard forward network cluster layouts, the goal is to minimize the area of the forward network cluster or bus shortest length. They are hard module layout issues. For the BBL mode and the gate sea mode of the game, when all the modules are hard modules, it is a layout problem; if some or all of the modules are soft modules, it is a planning problem.

RETRACTED

The network without hidden layer is similar to the linear regression model. The linear regression in Figure 6 can be regarded as a forward three-layer neural network without hidden layer, and the output neuron adopts a linear transformation function, such as the linear regression represented by *w*. The model can be expressed as a forward three-layer neural network with 5 independent variables and one output without hidden layer, and the output neuron adopts a linear transformation function, wherein the input value of the neural network is five and the deviation value, and the output value is *y*.

## 5. Application and Analysis of Optimization Model of Urban Cultural Space Construction Layout Based on Forward Three-Layer Neural Network

### 5.1. Forward Three-Layer Neural Network Data Extraction

The initial construction layout of the forward three-layer neural network is based on certain selection rules, and each time one or several forward network clusters are selected from the unplaced forward network cluster, according to their relationship with the placed forward network cluster *A*′. According to certain placement rules, they are placed in appropriate positions on the forward network cluster until all the unplaced forward network clusters have been placed, thus forming the initial configuration of the layout.

(11) $$\begin{array}{c} \frac{1-\exp\left(x,n\right)}{\exp\left(x\right)\exp\left(n\right)}-x\left(\frac{u\left(x\right)}{a},\frac{u\left(a\right)}{x}\right)⟶\frac{1-\exp\left(-ax/dx\right)}{\exp\left(-ax/dx\right)}. \end{array}$$

In constructing the layout, the forward network cluster positions are not moved once they are determined. At the same time, an initial layout is obtained only when the construction is complete. The initial navy needs to determine the selection function and placement rules to be used, so its algorithm consists of two parts: selection and placement. Selection is to select one or several forward network clusters from the set of unplaced forward network clusters to prepare for placement; placement is to place the selected forward network clusters in the appropriate positions of the forward network clusters. The initial layout should make both strategies (objective functions) consistent.

The degree of diversification is an important indicator reflecting the overall structure and completeness of regional cultural space layout types. The diversification of cultural space utilization can create a harmonious and friendly environment, enrich the lives of urban and rural residents, and reflect the essence of urban cultural space construction. This paper uses the Gibbs–Martin diversification index model to measure the degree of diversification of the types of cultural spatial distribution in regional urban circles. The value of GM in Figure 7 is between 0 and 1, 0 means there is only one type of cultural space layout, and the closer it is to 1, the higher the diversity of cultural space layout types in the region. The diversity index is affected by the number of cultural space layout types. When there are several cultural space layout types, the maximum value of GM is 1/*n*.

(12) $$\begin{array}{c} n\left(t\right)=\prod y\left(t\right)-1\prod y\left(t-1\right)-1\prod y\left(t-2\right)-1\prod y\left(t-n+1\right)-1. \end{array}$$

We take the sources and drains of the nets of all participating lines as points in the set. In order to calculate the dimension of the forward network cluster of the plane set *A*, we can construct some squares with side lengths of 6 or called forward network clusters, and then calculate the number of “forward network clusters” of different 6 values that intersect with *A*; this dimension is the logarithmic rate of increase of muscle (*A*) when 6-0, or it can be estimated by the slope of the graph with the function log*N t*(*a*) relative to a tog as shown in the text. In fact, since the points of set *A* are always limited, when 6 takes a smaller value, each point is included in a “forward network cluster,” which is nothing to choose a smaller one meaningful. On the basis of analyzing the influencing factors of land use structure change, the feedback relationship between them and the law of time series dynamic change are discussed, and the connection between them is represented by connecting symbols to form a closed loop, thus forming a causal relationship diagram.

RETRACTED

### 5.2. Simulation Realization of Urban Cultural Space Construction Layout

Use MATLAB language to construct the activation function of typical neural network, such as s-type, linear, and other activation functions, and write various subroutines for network design and training. Network designers can call the neural network design and training programs in the toolbox according to their own needs, so as to free themselves from tedious programming and improve development efficiency. Therefore, all the realizations of the cultural space layout planning model based on the forward three-layer neural network in this research are realized under the Windows operating system environment, and the visualization development tool of the layout MATLAB is realized.

There may be many planning objectives that need to be followed for the spatial planning of urban culture in Figure 8, such as minimizing urban traffic congestion, environmental pollution, maximizing economic benefits, and providing good infrastructure services, but in order to simplify the processing and considering the difficulty of data acquisition, this paper only considers two goals, namely, minimizing the cultural space development cost of the layout plan and maximizing the overall coordination of the layout plan in space, regardless of the road network layout. Space coordination is the degree of life comfort and production convenience. For example, school, entertainment, and commercial land should be close to residential land, and industrial land with environmental pollution should not be adjacent to residential land.

(13) $$\begin{array}{c} \left\{\begin{array}{c} \frac{\forall dp\left(t\right)}{d\left(t\right)}=1,\;dt\;>dp\left(t\right),\\ \exists r\left(t\right)-\frac{1}{r\left(t\right)}-\frac{p\left(t\right)}{dp}=1-tdt\;. \end{array}\right. \end{array}$$

When some forward network clusters of an inhibition *tl* can move to the left in the direction of the *X*-axis, it is called left compression. When some forward network clusters in a layout can move to the bottom edge in the *y*-axis direction, it is called bottom edge compression. When some forward network clusters in a layout can be compressed left and bottom, it is called left-bottom compression. For a given layout *P*, through a series of compressions in the *X* and *Y* directions, a corresponding left-bottom compression layout *P* can always be found.

### 5.3. Example Application and Analysis

Select 24 indicators with the concept of urban cultural space as the input vector, and the initial weight is a random number between [0, l]. Since the data of each indicator have different dimensions and units, the differences in their values are large, which will inevitably affect the results of the partition. Use the detection samples to test the learned neural network model, get the sample detection error, and judge whether the established model meets the requirements. If it does not meet the requirements, re-select the sample or set the learning parameters, and retrain the network until the network training is successful. This model adopts the standard deviation standardization; that is, the original data in Table 2 are normalized.

At the same time, in combination with the Terre law, the ecological quality of each cultural space layout type in the regional urban circle is assigned a value between [0, 1], which is defined as the relative ecological value of different cultural space utilization types, reflecting the different cultural space layout types per unit area for the proportional relationship between the ecological values. Among the types of cultural space layout in regional urban circles, the ecological value of forest land is the highest, and its relative ecological value is assigned a value of 1.000. The ecological value is adjusted to 0.305, the values of garden land, grassland, and other agricultural land are 0.925, 0.826, and 0.312, respectively, and the construction land (residential and independent industrial and mining land, transportation land, and water conservancy facility land) is unified. The value is 0.015, the ecological service function potential of the undistributed land needs to be developed, and the value is lower, which is 0.035.

(14) $$\begin{array}{c} \langle \begin{array}{c} b=a-a*\frac{\left(s\left(t,1\right)/s\left(1\right)-s\left(t,0\right)/s\left(0\right)\right)}{\left(1-a\right)},\\ a=a*\frac{s\left(t,1\right)}{s\left(1-a\right)}. \end{array} \end{array}$$

The change of urban cultural space layout is a complex process with multiple variables, multiple objectives, and the influence of multiple factors.

RETRACTED

If the network has not been successfully trained when the number of training times has exceeded the maximum number of training times, a back judgment check will be performed on the collected samples. Use the optimal network trained in Figure 9 to perform multiple sets of generalization predictions for Fr and vertical spacing a, where Fr = 0.3～0.7, set the step size to 0.02, a total of 20 groups, and the vertical spacing range *a* = −3.0*m* + 3.0*m*, and set the step length to 0.06 m, a total of 100 groups of cases. The total resistance value per unit displacement of the 2000 sets of flight states can be predicted by programming. Intuitively comparing the two graphs, the trend is consistent, indicating that the network simulation has a certain accuracy. However, there is a huge difference in calculation time between the forward three-layer neural network simulation and the CFD calculation simulation: it takes nearly a day for CFD to calculate the resistance corresponding to a set of Fr and a, and the larger the Fr, the longer the time. The process of grid division is more time-consuming and labor-intensive, while the training of the forward three-layer neural network takes only two hours, and the predicted 2000 sets of data only take a few minutes. It can be seen that the forward three-layer neural network model has strong nonlinear mapping ability, and its results can fully meet the requirements of engineering practicality through training.

RETRACTED

## 6. Conclusion

Due to its rapid economic development, relatively complete urban-type cultural space layout types in the old urban area, and a wide and balanced distribution of mixed-use areas in the suburban urban-rural integration zone and the types of agricultural land in the outer suburbs, the region has become the area with the most active changes in cultural space layout/coverage. This paper mainly constructs an objective function to evaluate the urban cultural space layout from various aspects, such as cultural space nonexpenditure cost, cultural space spatial coordination, land parcel shape compactness constraints, distance constraints, and direction constraints. Evaluation is a very important content in the preparation, approval, and implementation of cultural space layout planning. Regional cities have the highest diversity index of cultural space layout types, with a GM of over 0.771. Therefore, the optimization of urban cultural space layout is a typical multi-objective decision-making problem, and it is obviously unreasonable to take a single objective as its optimization direction. If the function is used to create an accurate network, the number of neurons in the hidden layer is automatically selected so that the error is 0, so there is no need to manually determine the number of neurons in the hidden layer. In general, the diversity index of cultural space layout types in regional urban circles shows a transitional trend from southwest to northeast. Therefore, on the basis of analyzing and comparing the deficiencies and problems of traditional evaluation methods, this paper designs the evaluation model of cultural space layout planning based on the forward three-layer neural network and proposes four effective methods for sample construction in the evaluation model of planning scheme. A standardized utility function for evaluating different types of planning schemes is designed. Taking the optimal evaluation of regional cultural space layout planning schemes as an example, a network structure is used to construct an empirical model for evaluating regional cultural space layout planning schemes.

## Figures and Tables

**Figure 1:** Nested flux distribution of forward three-layer neural network.

**Figure 2:** Analysis of neural network training process.

**Figure 3:** Feedforward network cluster of urban culture sample input.

**Figure 4:** Forward three-layer neural network interconnected two-dimensional array.

**Figure 5:** Evaluation of urban cultural data under the forward three-layer neural network.

**Figure 6:** Sector distribution of spatial construction layout index allocation.

RETRACTED

**Figure 7:** Forward three-layer neural network data objective function distribution.

**Figure 8:** The layout process of urban cultural space construction.

**Figure 9:** The optimal network of urban cultural space construction and layout.

**Table 1:** Results of spatial construction layout.

Spatial construction case	Planning *a*	Planning *b*	Planning *c*
Sample input	60.557	43.701	28.231
	46.237	11.765	10.822
	52.648	32.078	22.793

Sample output	2.258	48.341	27.410
	76.900	39.401	18.311
	10.942	46.608	32.279

**Table 2:** Algorithm steps of forward three-layer neural network.

Algorithm steps of network	Description text
# Placement 0, 0 would be the bottom left, 1	In the regional urban circle *dp*(*t*)
Ax.text2d (0.05, 0.95, “2D text,” transform)	The proportional relationship *dp*(*t*)/*d*(*t*)
# Tweaking display region and labels	Between the ecological *a∗s*(*t*, 1) values
Ax.set_xlim (0, 10)	Is assigned a value between [0, 1]
Ax.set_ylim (0, 10)	Reflecting the different cultural *s*(*t*, 1)/*s*(1)
Ax.set_zlim (0, 10)	Which *y*(*t* − 1) is defined
Xx = np.arange (−5, 5, 0.5)	Space layout types per unit imager(*i*, *j*).
Yy = np.arange (−5, 5, 0.5)	As the relative ecological value of *p*(*t*)/*dp*
*X*, *Y* = np.meshgrid (xx, yy)	Of each cultural *r*(*i*)*r*(*j*) space layout type
*Z* = np.sin(*X*) + np.cos(*Y*)	Different cultural space utilization types
Matplotlib.pyplot.scatter (*x*, *y*)	At the same time, the exp(*x*, *n*) quality

## Data Availability

The data used to support the findings of this study are included within the article.
